The article "Location-Dependent Query Processing: Semantic Cache for Real-Time Smart City Analytics" was retracted in 2023. Reasons: signs of a paper mill; compromised peer review; unreliable results or conclusions.

# Location-Dependent Query Processing: Semantic Cache for Real-Time Smart City Analytics

**DOI:** 10.1155/2021/9958647

**Published:** 2021-12-21

**Authors:** Rabia Hasan, Waseem Shehzad, Ejaz Ahmed, Hasan Ali Khattak, Ahmed S. AlGhamdi, Sultan S. Alshamrani

**Affiliations:** ^1^Department of Computer Science, National University of Computer & Emerging Sciences, Islamabad 45000, Pakistan; ^2^School of Electrical Engineering and Computer Science (SEECS), National University of Sciences and Technology (NUST), Islamabad 45000, Pakistan; ^3^Department of Computer Engineering, Collage of Computers and Information Technology, Taif University, P.O. Box 11099, Taif 21944, Saudi Arabia; ^4^Department of Information Technology, College of Computer and Information Technology, Taif University, P.O. Box 11099, Taif 21944, Saudi Arabia

## Abstract

With the advent of wireless sensor networks and their deep integration with the world have enabled users worldwide to achieve benefits from location-based services through mobile applications, the problems such as low bandwidth, high network traffic, and disconnections issues are normally extracted from mobile services. An efficient database system is required to manage mentioned problems. Our research work finds the probability of user's next locations. A mobile user (query issuer) changes its position when performing a specific mobile search, where these queries change and repeat the search with the issuer position. Moreover, the query issuer can be static and may perform searches with varying conditions of queries. Data is exchanged with mobile devices and questions that are formulated during searching for query issuer locations. An aim of the research work is achieved through effectively processing of queries in terms of location-dependent, originated by mobile users. Significant studies have been performed in this field in the last two decades. In this paper, our novel approach comprise of usage of semantic caches with the Bayesian networks using a prediction algorithm. Our approach is unique and distinct from the traditional query processing system especially in mobile domain for the prediction of future locations of users. Consequently, a better search is analyzed using the response time of data fetch from the cache.

## 1. Introduction

The role of a mobile computing in computer science is significant that is in information, computing, and telecommunication (ICT) domains. The ICT domain consists of wireless networks with the mobile devices. Pervasive mobile applications generate new opportunities and challenges in computing such as databases and networks. An excessive usage of mobile applications and services is related to hardware technologies and wireless network systems [1]. Wireless applications plays an important role in social networks [2], vehicular networks [3], healthcare informatics [4], financial tech, and cloud computing [5], by managing a connection between mobile database systems and servers. Data is exchanged using mobile devices whereby queries are generated and processed. A new search is emerged in the query processing domain. This study consists of two categories in which different queries are used to access the data. Normally, queries along with their results and data are mapped with the current locations of mobile users, such queries are called location-related or geolocation-based queries. Queries rely on location information, where the location is passed as a parameter. In location-dependent queries, the queries are transmitted with the change in locations (see Figure 1) [6].

A query consists of mobile client static object is managed in terms of client/user queries. For example, in query “where is the nearest restaurant?” there will be multiple locations or location may be changed. Since the client/node issues the query for mobile, execution of queries may extract irrelevant locations for the client in the new location. Moreover, the client may change the location and the query response is no longer required. After processing, the query results need to be validated in the first type of query as the query issuer's location can be changed, and the results may need calculation accordingly [7].

Various use cases can be elaborated to understand the above-mentioned challenge [8]. However, with the change in locations, the response may vary. The results of some query at one location may be different from the results of the same query at some other location. For instance, if the user queries about the moving objects without changing its own position, this type of query is called *static client mobile objects.* For example, another type of query would be “the number of all cars passed by a user”. Finally, when both user and objects are moving then query would be challenging to process as both the client and objects are moving continuously, and information of both user and objects needs to be stored [9]. When both user and objects are moving such query can be handled easily before the first two types of query problems are resolved.

Queries are location-aware in which location is already defined inside the query. For example, “the names of all hospitals in downtown” and “what is the distance to the airport from the main city?” Typically, these queries do not depend upon the location of the query issuer (user). If a user with a mobile is moving and repeating the query frequently, the result can be different because the user's location is changing [11]. The factor of processing the query is costly where communications are often difficult to measure when user with mobile devices is changing the location. The queries are called location-dependent queries (LDQ) [1, 10] in which geographic locations of users are important. Similarly, using semantic cache schema an algorithm is introduced for dividing the queries into probability and remainder queries [12]. LDQs are divided into three categories related to static and moving users and objects as shown in Figure 1.

Continuous queries are those which are answered frequently with the change in locations, mentioned inside the queries. In terms of mobile computing, such queries are processed with the asymmetric features of mobile devices' such as energy issues, low battery power, and less bandwidth. These features affect the processing of queries. Besides, servers keep records of locations of all mobile devices and need to be updated when a mobile user/client changes its position.

The purpose of this study is to adopt a mechanism that can predict and preprocess data to reduce the overall response time using a prediction system flow described in Section 3. The usage of a cache memory helps in producing results on the same next query issued by any mobile client. This means the minimum processing is performed in terms of improved response time.

Answering the LDQs will help in understanding the requirements in paper with the following key characteristics [12]:

- A query user can be located through general packet radio service (GPRS) before processing the query
- Keep track of the position of the user. Update the database each time when a user changes the location
- Location of user changes and database for location is updated. This keeps tracking of user's location
- Analyze and calculate the query results with the prediction of future information. For validating the query results, the time interval between submitting a query and sending results back is measured
- To process queries efficiently, technologies such as caching, indexing, and data replication are used
- The values of locations of users and prediction are not calculated correctly

The remaining paper is structured as follows: Section 2 describes the related studies. The motivation towards LDQ validations are covered in Section 3.  Section 4 illustrates Bayesian networks using a prediction algorithm. Implementation methods are discussed in Section 5.  Section 6 provides the experimental results followed by the conclusion in Section 7.

## 2. Related Work

Several issues and challenges in the processing of LDQs, e.g., communication cost, are difficult to measure when mobile devices change their locations. Location management performs two operations, i.e., Lookups and Update. The Lookups retrieves the user/client location, whereas the Update is needed in all sites in a mobile network. There are different updating methods, and any site can be updated that shares the updated location with all other sites. Moreover, each site, which increases the update cost, can be updated individually. To solve the problem of users' location information, the location binding method is used. The binding is managed by location-based services, which identify the location and bind it with the query. This gives rise to another problem of granularity mismatch [1].

A suitable query language needs to be developed to express the types of queries that include operators, e.g., *close to* and *within*. Caching is one of the techniques to solve the data management issues. Whenever a client changes its position, the data in mobile database systems remain no more valid. Therefore, caching is a technique through which we can check data validation, whereas through semantic caching, we can predict future results for further queries. Other limitations are low battery power, limited bandwidth, and frequent disconnections.

A semantic cache technique that stores data and its descriptions is proposed in [10]. It uses the Voronoi diagram to index data objects. The proposed method is used to retrieve the nearest neighbor queries. It can be assumed from the experiments that the client location and speed are known from the GPRS and query issue time stamp. A large area is divided into regions, and a *V*_*d*_ index is constructed for each of the service objects in the region. By measuring the client speed, the next nearest neighbor service is predicted. The cache contains the information of query regions (usually a circle) in which the client is the center of the circle, whereas the radius is the shortest distance. When a query is submitted, the data can be collected from the cache. Otherwise, the whole query is sent to the server. The results show the efficiency of this technique. However, when the number of service objects in a region increases, the cache hit ratio decreases. Moreover, if a client remains in the same region, all cached data is assumed to be valid. Nevertheless, as it moves to another region, the cache will be cleared and updated with the new data [11].

The drawback of the semantic cache was overcome by a technique presented in [12], wherein the authors have proposed a semantic cache schema, which supports processing different types of queries. It was based on the VCKNN query processing algorithm and the cache item structure that decides which data to be stored. They also defined a cache management algorithm to calculate which part of the query can be answered by dividing the query into two types, i.e., probe and remainder [13]. Through a cache replacement policy, cache items having a minimum number of references can be replaced. It works the same as the traditional LRU policy. They concluded that there should be a cache schema for the efficient utilization of the cache.

Grid-partition index has also been used to answer the nearest neighbor query using semantic and hybrid caches [14]. Some of the benefits of using cache in distributed systems are such that they are transparent for the application and do not affect the functionality of the application that utilizes a cache, as described in [13–16]. Unlike centralized systems, data is stored in the cache in webpages. The webpages give answers from a query called cache units and the query itself is a cache descriptor. The query containment problem is highlighted, i.e., the query text must be compared with cache descriptors to find the desired answer without evaluating the query. For experiments, the authors assumed a conservative algorithm that never produces false results. The algorithm also processes queries by extracting simple expressions from the incoming query and matches it with cache descriptors. Still, there is a need to provide such a database system that can predict and cache the most likely accessed data. Query processing must divide or break up a query to utilize the benefits of the cache [17].

Another study in [18] presents a semantic cache arrangement, where such arrangement accesses location-dependent destination (LDD) in mobile computing. Initially, a mobility model is used to represent mobile users' moving behaviors and properly define LDD. Then, query processing and cache management tactics are examined. Finally, the proposed approach is evaluated using a simulation study. The evaluation purpose was to check the semantic caching scheme's performance and its replacement strategy, named FAR. The results indicate that semantic caching is more flexible. LDD is more effective to be used instead of page caching. The performance of page caching is problematic to the database's physical organization. Moreover, the results also show that the semantic cache replacement strategy, i.e., FAR, is robust to various types of workloads. Additionally, the study also addresses the problems in building an abstract model of moving objects and formally defines the queries.

The authors in [10] present a scalable system based on mobile agents by supporting a distributed processing of LDQs in mobile environments [19]. The proposed system processes LDQs in a completely decentralized way without overloading wireless user devices. It caters to scenarios where users are issuing queries and other exciting objects are moving using a location prediction algorithm. Moreover, it is well adapted to environments where location's data is distributed in a network and processing tasks can be performed in parallel. This way it allows high scalability. A mobile agent can be incharge of tracking the location of interesting moving objects and refreshing the answer to a query efficiently. The system is evaluated through an experiment by carrying out simulations of a sample scenario.

The authors in [20] discuss that how mobile devices have captured the entire world's coverage, leading to the demand for location-based services and applications used in daily routines. Location detection capability services constitute a significant part of mobile devices. The paper discusses an environment where mobile objects have no capability for location detection, and location-aware mobile sensors are scattered for sensing mobile devices' presence. A sensor can only detect and identify those mobile objects lie in their range but cannot identify their exact locations. The sensor readings are aggregated and sent to the server at regular intervals. The system supports mobile LDQs over mobile objects.

Approximate Moving Range (AMR) query is presented in [11], which is a new class of location-based query that introduces a probabilistic technique for processing AMR. The environment is based on mobile sensors, where each sensor is modeled as a moving rectangle representing its sensing range. Each sensor can detect unaware location objects discovered in its range. The AMR query pointed at moving objects with no capability of location detection. The database server can evaluate the AMR queries based on the detection of mobile sensors on moving objects. The proposed query was tested on different simulation studies to evaluate its processing technique. The results showed that the AMR query processing technique is very efficient and reliable. It is also highly cost-effective and scalable than standard approaches.

In [19], the authors discuss that how mobile devices have made significant advances, providing their users with outstanding services. The study proposes a system that deals with mobile environments and supports the processing of continuous LDQs. This research includes a new approach for continuous LDQs in a wireless environment with decentralized solutions for continuous moving queries. The system was based on tracking related moving objects with the help of mobile agents. When a user enquires a query in the system, the answer is refreshed after a certain period, and the network of agents adjusts itself to provide data as new as possible.

The system's main features include the following: (1) a flexible and distributed architecture is required that could be scalable when the number of moving objects and proxies increases in specific scenarios. For a considerable number of moving objects, the centralized approach is not feasible. (2) To avoid wireless user devices with overloading processing tasks, queries were performed on proxies and fixed networks instead of wireless networks. (3) Any object in the scenario can access the location query. (4) Query answers are continuously updated and selected by a user because the location data is changing dynamically. The proposed system's main advantage is a general solution for processing LDQs for users enquiring any query. Besides, the system is efficient concerning processing continuous queries. Moreover, it is adaptable to environments where data location is distributed over a network providing scalability to the system and optimizing wireless communications.

In [21], a scheme is proposed that provides a comprehensive study on mobile database systems, their characteristics, and architecture for query processing in mobile databases. Apart from describing the existing architecture challenges, the authors have investigated the location privacy protection concerns associated with mobile database query processing. Mobile database systems are generally considered as an extension of distributed database systems but differ in terms of mobile environments' constraints. The constraints involve power restriction and frequent disconnections. Other fundamental problems are significantly associated with mobile database systems, i.e., scalability (low bandwidth is covering long transactions). Based on query processing, mobile database systems have three layers, i.e., the Application layer, the Middleware layer (query, cache, network), and the Database layer. The best noticeable technique in the context of location privacy for LDQs is *K*-anonymity. However, privacy concerns are still an open area of research as a little study has been accomplished to produce efficient algorithms. There is also a need to empirically evaluate the results of existing techniques in this context.

The focus is to study the challenges and issues faced by LDQ processing [22]. Location-based queries can be classified into spatial queries or temporal queries, which can be further categorized into continuous or noncontinuous queries. Range queries include the objects lie within a specific region, while nearest neighbor queries include the objects lie closer to a specific region. Navigation queries provide the path to users in a specific location. In this paper, different methods for LDQs and the problems faced in the data management system have been discussed. Some challenges are also possible in mobile systems in terms of data management. The methods presented to solve the issues are caching and broadcasting data. Caching techniques make accessing data fast and lesser the network traffic caused by processing the LDQs. Broadcasting of data means transferring information to a large number of users over a mobile network. One method is such that the server broadcasts the invalidation report, while the other is that every mobile device receives the updated data if its value is changed on the server. There is a local database between a mobile and the central server that acts as a mediator.

In [23], the authors propose a query formalization technique that uses both location-dependent and location-independent query models. It provides a general view of location-related queries. It also distinguishes between location dependence and location independence. The proposed approach provides implicit translation of both LDQs and location-aware queries. Moreover, a software architectural style, named Location Dependent Services Manager (LDSM), is also proposed. This architecture aims to aid in the translation process.

Many personalized techniques have been widely studied that use the auto recommendation system [24]. Mobile systems provide location-based services to users based on their physical locations. In this paper, a recommendation system has been built, which is map-based to overcome all the abovementioned problems. Mobile users face problems due to small screens and interfaces of mobiles. This technique improves the interface system. Old recommendation systems use collaborative filtering, i.e., similar users have similar interests. This research uses a map-based interface close to user familiarization to overcome the issues of visualizing and resource usage of mobile devices. Today, people face many problems in utilizing navigation services due to mobiles' bad interfaces and low usage of resources. The presented system collects the information, time, location, and weather of the user's physical location and recommends the desired result in the form of a map. The study presented the BN-based recommendation system, which reflects the user's recommendation using information from mobile devices user profiles.

In [25], a novel approach has been proposed to enhance and extend Location Base Service (LBS)'s privacy to users. Information was extracted from LBS queries with regards to service providers. Authors have developed and evaluated MobiCrowd, a scheme that enables LBS users to hide in the crowd and reduce their exposure while continuing to receive the location context information they need. MobiCrowd achieves this by relying on the collaboration between users who have the incentive and the capability to safeguard their privacy. In this study, a novel analytical framework is proposed to quantify the location privacy of distributed protocol. The epidemic model captures the hiding probability for user locations, i.e., the fraction of times when the adversary does not observe user queries due to MobiCrowd. In this model, the Bayesian inference attack estimates the location of users when they hide. The extensive combination of epidemic and Bayesian analysis elaborates a significant improvement across both individual and average mobility prior knowledge scenarios for the adversary.

The authors in [26] propose a semantic cache schema to extend the domain of query types. Semantic cache schema answers all types of queries based on the query graph model and query conversions to QGM. Semantic cache schema, data structure of cache items, cache management algorithm, and cache items replacement algorithm are designed by planning the semantic cache schema. The semantic cache schema gains significance in performance, while other methods are evaluated using simulations. Response time, data volume transferred from the server, and the number of connections to the server are the performance parameters that were measured and compared significantly. The performance is typically expected when submitted queries are more dependent on each other semantically. An application domain extends and broads in mobile systems with the study of elimination of this environment's limitations. There are several semantic cache schemas developed with simple query types. There is a need for a semantic cache schema that can answer all queries as a complete solution.

## 3. Motivation

A mobile user/client is in region R1, and queries are about object1. The results of query1 are stored in the local cache. Now, when a user changes its location from regions R1 to R3 and generates the same query, the data stored in the cache remains no more valid, as the query needed to be answered according to its current location. So, we must send the query again to the server to process, gather the desired data, and store it in the cache. As mentioned earlier, results are needed to be validated in LDQs whenever the user changes its location.  Figure 2 depicts this problem in a simplified way.

To utilize the cache to benefit us in reducing the network traffic and decrease the response time, we propose a technique that can predict the future location, prefetch the data, and store it in the cache. The flowchart presented in Figure 3 describes the working of the proposed system. This helps in evaluating the response time when the data of queries is saved in the cache.

Location server tracks mobile users and records their history based on their locations. All locations covered by a mobile client are recorded and saved. Whenever a client issues any LDQ, the database system will send the desired result to the mobile host and the future prediction of the user's next coming location. The predicted data will be stored on a local cache, i.e., a mobile host cache. The prediction of the user's next location maybe based on data classification and prediction algorithms. When a mobile client issues the next query, its results will be calculated from the cached data if the prediction is accurate and there will be no need to send the query to the server. It will be useful to use semantic cache for storing both query text and data.

There is a possibility that the future location's prediction of a user is false if a mobile client moves towards the new location which was never stored in the history. Therefore, we can predict the results based on history or patterns of issuing query of other mobile clients in that region.

## 4. Location Prediction Using Bayesian Networks

The proposed technique manages the primary database system and describes the work performed on mobile database systems in the query processing. To reduce the workload and processing on mobiles, it is highly recommended in this research that the minimum processing should be managed on mobile devices, keeping in view their issues, i.e., low bandwidth and limited battery. The proposed method's main idea is to examine the users' moving patterns according to the service objects. For this purpose, the history of users will be recorded to train the system. The prediction of the user next locations will be based on their current locations and the queried objects.

The central part of the processing has been diverted to the primary database system. Since our goal is to improve the response time, some modifications were also needed on the server side for this purpose. The proposed technique has utilized the Bayesian network to reduce processing time. All the locations and service objects related to their locations are stored in tables on the DBS server. Using Bayesian network, all tables containing information of service objects according to their locations are converted into conditional probability tables (CPT).

The Bayesian network has two components, i.e., structure and parameters. The structure includes directed ayclic graphs (DAG) while the parameter is a set of CPT, as presented in Figure 4.

It is imperative to note that this research focuses only on one type of LDQ, i.e., mobile client static objects. When moving from loc*_i_* to loc*_j_*, the object always remains the same, but location can vary from loc_i_ where *i* = 0, 1, 2, 3, ⋯*n*. Only the next location of the user will be predicted. For example, if a user is in loci and queries about “find the nearest hotel,” then only the user's next possible location will be predicted, wherein the object is always “hotel.” The query for processing and prediction remains the same until the user submits the query with different service objects.  Figure 5 shows prior probabilities of nodes *A* and *B*.

Algorithm 1 describes the proposed technique in a simplified fashion.

## 5. Implementation

All nodes shown in Figure 4 are dependent based on location and the object queries. To predict the next location, we calculate the posterior probabilities. For any dependent node (location), we can calculate the probability as follows:

If the next possible location of the user is Hi, where *i* = 1,2,3 ⋯ *n*, then

(1) $$\begin{array}{c} P\left(\text{Hi}\;|\;A\right)=\frac{P\left(A\left|\text{Hi}\right)P\left(\text{Hi}\right)\right)}{P\left(A\right)} \end{array}$$

The following example shows to understand that how the prediction can be performed at run time. In a region, the user is currently at location *A* and queries about object O1. The query processing process is defined in the following steps:

(i) On a mobile database system, the query can be evaluated whether it may be answered through cache or not. If the results are obtained, the query can be processed on a mobile system and no data will be sent to the server side
(ii) In other cases, if the cache does not hold the valid data, the query can be sent to the server along with the user's current location, which the location manager can determine
(iii) The database system will generate the desired result on the server side and, in parallel, the data may be evaluated using a Bayesian network
(iv) The user is at location *A* and queries about object *X*. The probability of moving to the next location *C* will be as follows:
  (2) $$\begin{array}{c} P\left(C\;|\;X\right)=\frac{P\left(C\left|Xi\right)P\left(Xi\right)\right)}{P\left(C\right)}. \end{array}$$

Similarly, the probabilities of the dependent nodes can be calculated, and the next location may be selected with the highest probability as follows:

- The server will now send back the results along with the predicted data
- On receiving, a mobile device will show the output, and the prefetched data can be resided in the cache to answer the next query
- As soon as the user changes its location from *A* to any other one, the previous data will be no more valid. According to the moving speed of the user, mobile D.B. regenerates the query for the new location. The new query will again match with the cache descriptors to get the results
- If the prediction is accurate, a signal will be sent to the server to notify it, where all the values of CPTs will be updated

## 6. Discussion

Figure 6 represents two different graph locations, which use datasets in the Weka tool. At the same time, the similarity probabilities are shown in Figure 7.

Figure 7 shows all locations, named *A*, *B*, *C*, *D*, and *E*, within the city. The arrows in the graph show the roads between two locations. If a user is at location *A* and moves from *A* to *B*, then we have its previous and current locations saved as a given probability, and the user's next location may be predicted, which can be either *C* or *B*. The probability of moving to location *C* is known as posterior probability, which a Bayesian network will predict.

Table 1 has two attributes, i.e., previous, and current location. With the help of these, we will predict its next location (class attribute). The actual dataset has 100 instances, which we used for training and testing of the Bayesian network. Four datasets are presented for graph 1, while two are displayed for the graph in Figure 7. Following is an example of how it works in a Bayesian network. First, we will compute the required probabilities from the given dataset. Next, these probabilities help us predict the user's next moving location to *C*, given *A* and *B*. According to the predicted location, the following location data will be prefetched and saved in the cache.  Table 2 depicts both graphs' mean future-based probability with datasets. Thus, for mobile P2P services, we have observed that the range queries have shown incremental progress while performing the query results [27].

## 7. Conclusion

The processing of Location-Dependent Query (LDQ) processing has been more challenging considering the massive increase in the usage patterns shifting massively towards mobile clients. Hence, there is always a need for an efficient prediction algorithm that can determine accurate results based on context. This will also provide better performance concerning time complexity for more extensive databases. For this purpose, this study focuses on predicting the future based on the history of mobile users. The Bayesian network's help has made it possible to manage LDQs to be processed in minimum time, as searching and prediction can be administered faster than the traditional database systems. In mobile P2P services, the range queries are used for messages by performing query results incrementally. This research work has limitations in not managing the case when both client and objects move their locations together. The more the system is trained, the more the chances of the algorithm is accurate when the data availability is managed effectively.

## Figures and Tables

**Figure 1:** Classification of location-related queries.

**Figure 2:** Mobile client static objects.

**Figure 3:** Flowchart of the proposed system.

**Figure 4:** Directed acyclic graph.

**Figure 5:** (a)–(c) show the prior probabilities of node *A* and node *B*, which represent locations in a region. (c) shows the posterior probabilities (missing values) that are yet to be calculated.

**Figure 6:** Sample graph 1 for datasets.

**Figure 7:** Sample graph 2 for datasets.

**Algorithm 1:** Query processing using semantic cache.

**Table 1:** Data set with three types of locations.

Previous location (given)	Current location (given)	Next location (prediction)
*A*	*B*	*C*
*B*	*C*	*D*
*C*	*D*	*E*

**Table 2:** Results of two graphs using Weka tool.

DATASETS	GRAPH #1	GRAPH #2
Dataset 1	68.80%	86.69%
Dataset 2	76.00%	87.88%
Dataset 3	77%	Not available
Dataset 4	70.80%	Not available

## Data Availability

The data for this research is incorporated in the manuscript.

## References

[1] Mäkelä L., Boedeker M., Helander N. (2020). Value emergence in the usage of mobile news alerts. *Digital Journalism*.

[2] Masood F., Ammad G., Almogren A. (2019). Spammer detection and fake user identification on social networks. *IEEE Access*.

[3] Tayyaba S. K., Khattak H. A., Almogren A. (2020). 5G vehicular network resource management for improving radio access through machine learning. *IEEE Access*.

[4] Hameed A. R., ul Islam S., Almogren A., Khattak H. A., Din I. U., Gani A. B. (2020). Towards energy-efficient mobile ad optimization: an app developer perspective. *Applied Sciences*.

[5] Malik F. M., Khattak H. A., Almogren A., Bouachir O., Din I. U., Altameem A. (2020). Performance evaluation of data dissemination protocols for connected autonomous vehicles. *IEEE Access*.

[6] Kottkamp H. E., Zukunft O. Location-aware query processing in mobile database systems.

[7] Judge M. A., Manzoor A., Khattak H. A., Din I. U. (2020). Secure transmission lines monitoring and efficient electricity management in ultra-reliable low latency industrial Internet of Things. *Computer Standards & Interfaces*.

[8] Thomas D., Thampi S. M. (2011). Mobile query processing-taxonomy, issues and challenges. *International Conference on Advances in Computing and Communications*.

[9] Khattak H. A., Tehreem K., Almogren A., Ameer Z., Din I. U., Adnan M. (2020). Dynamic pricing in industrial internet of things: Blockchain application for energy management in smart cities. *Journal of Information Security and Applications*.

[10] Zheng B., Lee D. L. (2001). Semantic caching in location-dependent query processing. *International Symposium on Spatial and Temporal Databases*.

[11] Seydim A. Y., Dunham M. H. (2005). Location-dependent query processing benchmark. *Wireless Information Highways*.

[12] Safaei A. A., Mallah M., Abdi F., Behjati S. (2011). Semantic cache schema for Continuous k-NN Queries in Mobile DBSs. *Information Technology Research Journal*.

[13] Novikov B., Pigul A., Yarygina A. A performance analysis of semantic caching for distributed semi-structured query processing.

[14] Naz S., Naeem M., Qayyum A. (2013). Performance evaluation of index schemes for semantic cache. *International Journal of Information Technology and Computer Science (IJITCS)*.

[15] Nascimento M. A., Alencar R. A., Brayner A. Optimizing query processing in cache-aware wireless sensor networks.

[16] Lee J., Eom Y., Sussman A., Nam B. (2012). DEMB: Cache-aware scheduling for distributed query processing. *Workshop on Job Scheduling Strategies for Parallel Processing*.

[17] Ardelius J., Grönvall B., Westberg L., Arvidsson A. A. On the effects of caching in access aggregation networks.

[18] Ren Q., Dunham M. H. Using semantic caching to manage location dependent data in mobile computing.

[19] Ilarri S., Mena E., Illarramendi A. (2006). Location-dependent queries in mobile contexts: distributed processing using mobile agents. *IEEE Transactions on Mobile Computing*.

[20] Petkova A., Hua K. A., Aved A. (2009). Processing approximate moving range queries in mobile sensor environments. *International Conference on Computational Science and Engineering*.

[21] Tarafdar M., Haghjoo M. S. Location privacy in processing location dependent queries in mobile database systems.

[22] Tabassum K., Hijab M., Damodaram A. Location dependent query processing–issues, challenges and applications.

[23] Seydim A. Y., Dunham M. H., Kumar V. An architecture for location dependent query processing.

[24] Park M. H., Hong J. H., Cho S. B. (2007). Location-based recommendation system using Bayesian user's preference model in mobile devices. *Ubiquitous Intelligence and Computing*.

[25] Shokri R., Theodorakopoulos G., Papadimitratos P., Kazemi E., Hubaux J. P. (2014). Hiding in the mobile crowd: locationprivacy through collaboration. *IEEE Transactions on Dependable and Secure Computing*.

[26] Safaeei A. A., Haghjoo M., Abdi S. Semantic cache schema for query processing in mobile databases.

[27] Lim J., Bok K., Yoo J. (2020). An efficient continuous range query processing scheme in mobile P2P networks. *The Journal of Supercomputing*.

